The article "Clove Buds Essential Oil: The Impact of Grinding on the Chemical Composition and Its Biological Activities Involved in Consumer's Health Security" was published in 2021. Journal: Biomed Res Int.

# Clove Buds Essential Oil: The Impact of Grinding on the Chemical Composition and Its Biological Activities Involved in Consumer's Health Security

**DOI:** 10.1155/2021/9940591

**Published:** 2021-08-02

**Authors:** Dorsaf Ben Hassine, Salma Kammoun El Euch, Rami Rahmani, Nessrine Ghazouani, Rouguiata Kane, Manef Abderrabba, Jalloul Bouajila

**Affiliations:** ^1^Laboratory Materials, Molecules, and Applications, IPEST, Carthage University, BP 51, La Marsa, Tunisia; ^2^National Agronomic Institute of Tunisia, Food Industries Department, Carthage University, Tunisia; ^3^Laboratory of Structural Organic Chemistry, Synthesis and Physicochemical Study, Faculty of Sciences of Tunis, El Manar University, Tunis, Tunisia; ^4^Research Unit of Valorisation of Active Biomolecules, Higher Institute of Applied Biology Medenine, University of Gabes, 4119 Medenine, Tunisia; ^5^Department of Life Sciences, Faculty of Sciences of Gabes, University of Gabes, Gabes, Tunisia; ^6^Laboratoire de Génie Chimique, UMR 5503, Université de Toulouse, CNRS, INPT, UPS, Toulouse, France

## Abstract

This study is aimed at identifying the chemical composition of the essential oil extracted from the *Syzygium aromaticum* seeds, as well as investigating its biological activities, insecticide effect, and allelopathic properties. The extraction yield was about 14.3 and 7.14% for grounded and ungrounded seeds, respectively. The GC-MS analysis allowed the identification of 17 heterogeneous compounds, including eugenol (68.7-87.4%), as major compound, cyperene (20.5-7.2%), phenethyl isovalerate (6.4-3.6%), and *cis*-thujopsene (1.9-0.8%), respectively, for grounded and ungrounded seeds. Concerning the antibacterial activity, the diameter of the inhibition zone reached 35 mm when the essential oil extracted from grounded seeds was applied against *Escherichia coli*. Regarding the antioxidant activity *via* the DPPH radical scavenging test, the IC_50_ varied from 1.2 ± 0.1 to 2.8 ± 0.5 *μ*g/mL. With respect to reducing power, the efficient concentration EC_50_ ranged from 32 to 50 *μ*g/mL. The essential oil exhibited also an allelopathic effect against seeds of *Hyoscyamus niger*, as well as an insecticide effect against *Sitophilus oryzae* with a DL_50_ value of 252.4 *μ*L/L air. These findings enhance the use of this spice as a natural food preservative and encourage its use in several fields, including pharmaceutical, cosmetics, agriculture, and therapy, that could be a strategic way to guarantee the consumer's health.

## 1. Introduction

Over the last decades, the use of aromatic plants for traditional medicinal purposes has gained a great interest. Thus, the Arab and Egyptian civilizations have attributed their use to religious recommendations [1]. Thereafter, the healing properties of extracts and essential oils were discovered and became common remedies to traditional medicines. For example, during the great epidemics in ancient Greece, the odorous principles of certain aromatic plants were spread by fumigation in the city streets to prevent the spread of infectious diseases. Fumigation of sick people is indeed one of the oldest therapeutic techniques [2].

The article "Clove Buds Essential Oil: The Impact of Grinding on the Chemical Composition and Its Biological Activities Involved in Consumer's Health Security" was published in 2021. Journal: Biomed Res Int.

Nowadays, modern medicine uses the therapeutic properties of essential oils and their constituents. Actually, many volatile compounds are common ingredients of pharmaceutical preparations. Thymol is used in dental care for its antiseptic properties, and eugenol is recommended due to its analgesic effect [3]. In an attempt to find new treatments to current diseases (cancer, asthma, Alzheimer, etc.), the scientific community has recently focused on the constituents of essential oils, thanks to the higher significant number of volatile compounds, such as sesquiterpenes, which showed remarkable pharmacological activities against diseases, in particular cancer [4]. Moreover, essential oils are used as natural antimicrobial, antioxidant, and bioactive agents against many pathogens [5].

*Syzygium aromaticum*, also called clove, is a dried flower bud, which belongs to the Myrtaceae family. This species is indigenous to the Maluku islands in Indonesia, and it is the most important and second valuable spice in world trade [6]. Clove bud essential oil is known for its antioxidant, antifungicidal, anticarcinogenic, and anesthetic activities and for its antiprotozoal effects, thanks to its richness in many phytochemicals, such as sesquiterpenes, monoterpenes, hydrocarbons, and phenolic compounds [7, 8].

Several researchers have reported the antibacterial activity of the essential oil from clove buds against different food-borne pathogens [9, 10]. However, to the best of our knowledge, current studies did not take into account the antigerminative effect of this essential oil, and neither did they take into account its insecticide power nor the effect of the size of the plant material on the essential oil chemical composition. All of these traits were the main objectives of this work.

## 2. Materials and Methods

### 2.1. Taxonomy and Preparation of Clove Buds

According to the US National Plant Germplasm System, *Syzygium aromaticum* (*S. aromaticum*) (synonym: *Eugenia cariophylata*), commonly known as clove, belongs to the Myrtaceae family, subfamily of Myrtoideae and Syzygiae tribe. It is a median-sized tree (8-12 m) native from the Maluku islands in east Indonesia [11]. It is an evergreen plant, with large leaves and terminal grouped flowers. These latter are initially pale in tint, and then progressively become green, before acquiring a brilliant red hue when harvested at 1.5-2 centimeters long. They are composed of a long calyx, which ends in four extended sepals, and four nonopened petals forming a small central ball. Clove buds were purchased from a local market in Kef (North-west of Tunisia). The buds were cleaned, sorted, and homogenized. The initial particle size for ungrounded buds was about 2 cm. Grounded buds had a size of about 0.6 mm. Two batches were prepared (ungrounded and grounded). Each one is composed of 50 g raw material. The samples were ground using an electric grinder (Moulinex AR 1105, France).

The article "Clove Buds Essential Oil: The Impact of Grinding on the Chemical Composition and Its Biological Activities Involved in Consumer's Health Security" was published in 2021. Journal: Biomed Res Int.

### 2.2. Hydrodistillation

Both grounded and ungrounded buds were subjected, separately, to hydrodistillation during 6 h using a Clevenger-type apparatus. The raw material was directly submerged in 500 mL distilled water in a round bottom flask (1 L capacity) containing a few pumice stones to regulate boiling. The entire extraction method was operated at atmospheric pressure. This technique consists of boiling the mixture, then condensing the vapors that are released using a water condenser. The condensation of this vapor mixture causes its separation into an organic phase, called essential oil, containing the majority of the odorous compounds, and an aqueous phase, called aromatic water, which contains very few odorous compounds. As the density of clove bud essential oil (1.062) at 20°C was superior to the water density (1.00), the separation of the organic and aqueous phases was a little bit difficult. In fact, the organic phase was below the aqueous one. For this purpose, the distillate was placed in a decanter. Salt-saturated water was then added. After shaking and degassing, the mixture was decanted. This step, called release, allows the separation of the essential oil from the aqueous phase, since the essential oil is less soluble in salt water than in water. The obtained essential oil was then recovered with the help of the decanter. After that, it was dried with Na_2_SO_4_ and stored in amber-colored bottles at 4°C for subsequent analysis. The Na_2_SO_4_ was removed by filtration of the EO. The extraction yield was calculated as follows:

(1) $$\begin{array}{c} \text{Yield }\left(\%\right)=\frac{\left(\text{EOV}*100\right)}{\text{DM}}, \end{array}$$

where DM is dry matter (mg), EOV is essential oil volume (mL).

### 2.3. Gas Chromatography and Gas Chromatography Coupled with Mass Spectrometry (GC-MS)

The identification of volatile compounds from *S. aromaticum* bud essential oil used the procedures of Ben Hassine et al. [5]. Analytical gas chromatography was carried out on a Varian Star 3400 (Les Ulis, France) Cx chromatograph fitted with a fused silica capillary DB-5MS column (5% phenyl-methyl-polysiloxane, 30 m × 0.25 mm; film thickness: 0.25 *μ*m). The analysis was performed using the following temperature program: temperature rise from 60°C to 260°C with a gradient of 5°C/min and 15 min isotherm at 260°C. A second gradient was applied to 340°C at 40°C/min. The injection volume was 1 *μ*L in 1 : 10 split mode. The carrier gas was helium with a flow rate of 1 mL/min. Injector temperature was held at 200°C. The mass spectrometer (Varian Saturn GC/MS/MS 4D) was adjusted for an emission current of 10 *μ*A and electron multiplier voltage between 1.400 and 1.500 V. Trap and transfer line temperatures were 220°C and 250°C, respectively. Mass scanning was from 40 to 650 amu. The identification of the oil constituents was based on a comparison of their retention indices (RI) relative to C_5_-C_24_ n-alkanes with those of the literature or with those of authentic compounds available in our laboratory. Further identification was made by matching their recorded mass spectra with those stored in NIST 08 and other published mass spectra. The percentage composition of the essential oil was calculated by the normalization method from the GC peak areas, assuming identical mass response factor for all compounds.

The article "Clove Buds Essential Oil: The Impact of Grinding on the Chemical Composition and Its Biological Activities Involved in Consumer's Health Security" was published in 2021. Journal: Biomed Res Int.

### 2.4. Free Radical Scavenging Activity: DPPH^•^ Assay

Spectrophotometric measurements were assessed according to the method of Ben Hassine et al. [5]. A volume of 1.5 mL essential oil dilution was added to 1.5 mL of DPPH^•^ solution (0.2 mM). After 30 min of incubation at room temperature, the absorbance was measured at 520 nm. The DPPH^•^ inhibition percentage (IP) was expressed as follows: IP(%) = ((*A*_blank_ − *A*_sample_)/*A*_blank_)∗100. Here, *A*_blank_ is the absorbance of the control containing only the solvent and DPPH^•^ solution. Radical scavenging activity was expressed in terms of IC_50_ (*μ*g/mL), and BHT was used as standard. IC_50_ represents the concentration at which clove EO exerts half of its maximal DPPH^•^ inhibitory effect. It indicates how much EO is needed to inhibit the radical by half, thus providing a measure of potency. A lower value of IC_50_ indicates more potent inhibitors. All measurements were replicated three times.

### 2.5. Ferric-Reducing Antioxidant Power: FRAP Assay

Experiments were done according to Kammoun El Euch et al. [12]. One mL of *S. aromaticum* essential oil was mixed with 2.5 mL of sodium phosphate buffer (0.2 M; pH = 6.6) and 2.5 mL of 1% K_3_Fe (CN)_6_. The whole mixture was incubated in a water bath at 50°C for 20 min. Then, 2.5 mL of a 10% TCA solution was added to the mixture, which was centrifuged at 6500 rpm for 10 min. The supernatant (2.5 mL) was then mixed with 2.5 mL of distilled water and 0.5 mL of a 0.1% FeCl_3_ solution. The intensity of the blue-green color was measured at 700 nm, and BHT was used as a positive control. The IC_50__%_ value (*μ*g/mL) is the effective concentration at which the absorbance was 0.5 for reducing antioxidant power and was obtained by interpolation from linear regression analysis. All measurements were replicated three times.

The article "Clove Buds Essential Oil: The Impact of Grinding on the Chemical Composition and Its Biological Activities Involved in Consumer's Health Security" was published in 2021. Journal: Biomed Res Int.

### 2.6. Antimicrobial Activity

The antimicrobial activity of clove buds essential oil was achieved according to the disc diffusion method [5]. Three types of Gram-positive bacteria (*Staphylococcus aureus* ATCC 6538, *Listeria monocytogenes* FMCC B-128, and *Bacillus cereus* ATCC 168) and two Gram-negative types (*Escherichia coli* ATCC 35150 and *Salmonella enteritidis* ATCC 13076) were used. A suspension of the tested microorganism (0.1 mL of 10^8^ cells per mL) was spread on nutrient agar. The discs have a 6 mm diameter, and against each microbial strain, one dose each of 1, 5, and 10 *μ*L of pure EO was applied to each disc, respectively, and separately, by injecting and placing on the inoculated plates. Penicillin (P), chloramphenicol (C), gentamicin (GM), and erythromycin 500 (E) were used as standard antibiotics to determine the sensitivity of the bacterial species tested. These plates, after staying at 4°C for 2 h to allow the diffusion of volatile compounds inside the Petri dishes, were incubated for 48 h at 37°C. Antimicrobial activity was evaluated by measuring the inhibition zone diameter (IZD) (mm) against the tested microorganism. The strain's sensitivity was evaluated according to IZD (*Ф*) as follows: (-) 6 mm < *Ф* < 10 mm: the strain is insensitive to the EO action; (+) 10 mm ≤ *Ф* < 15 mm: the strain is sensitive; (+ +) 15 mm ≤ *Ф* < 20 mm: the strain is very sensitive; (+ + +) *Ф* > 20 mm: the strain is extremely sensitive to the EO action.

### 2.7. Allelopathic and Insecticidal Effects

In light of previous results, tests for the allelopathic and insecticidal effects were carried out with the grounded clove bud essential oil, since it was responsible for the highest biological activity results.

#### 2.7.1. Allelopathic Effect

The allelopathic effects of clove EO on *H. niger* germination was tested following the method adopted by Zahed et al. with slight modifications [13]. Five concentrations (1, 5, 10, 20, and 30 *μ*L/mL) were used. Essential oil was diluted in 1‰ MeOH. Distilled water served as the control. Whatman No. 2 filter paper was placed in 9 cm diameter Petri dishes moistened with 5 mL of EO solutions. Five replications of 25 seeds were used for each treatment. To prevent evaporation, Petri dishes were sealed with parafilm and placed in an incubator at 25°C in the dark. After 10 days, the number of germinated seeds was recorded and the percentage of germination was calculated using the following formula:

(2) $$\begin{array}{c} G\;\left(\%\right)=\left(\frac{n}{N}\right)*100, \end{array}$$

where *n* is the number of germinated seeds in the test solution, and *N* is the total number of seeds. Seeds showing radicle emergence (2 mm) were recorded as germinated.

The article "Clove Buds Essential Oil: The Impact of Grinding on the Chemical Composition and Its Biological Activities Involved in Consumer's Health Security" was published in 2021. Journal: Biomed Res Int.

#### 2.7.2. Insecticide Effect

*(1) Insect Rearing*. *Sitophilus oryzae* adults were obtained from cultures initiated in the Laboratory of Materials, Molecules, and Applications at IPEST, La Marsa, Tunisia. Corn (*Zea mays*) seeds were used as a host. Insects were reared in darkness at 25°C in a relative humidity (R.H.) of 65 ± 5% and 16/8 (L/D) photoperiod. The old adult insects (7-10 days) were used for fumigant assay.

*(2) Fumigant Assay*. Fumigant toxicity assay of *S. aromaticum* essential oil was evaluated using the method described by Bachrouch et al. [14]. Two-centimeter-diameter filter papers (Whatman No. 1) were impregnated with the tested EO doses. The impregnated filter papers were then attached to the screw caps of 44 mL plexiglas bottles. Caps were screwed tightly on the vials; each one contained *S. oryzae* adults (1–7 days old). When no leg or antennal movements were observed, insects were considered dead. To evaluate the insects' mortality, amounts of 2.5, 5, 7.5, and 10 *μ*L EO from clove grounded buds, corresponding to concentrations of 41.7, 83.3, 125, and 166.7 *μ*L/L air, respectively, were prepared. Control insects were kept under the same conditions without any EO, and each dose was replicated three times. The number of dead and alive insects in each bottle was counted 24 h after initial exposure. The mortality was evaluated by direct hourly observation of the insects. Probit analysis [15] was used to estimate LC_50_ and LC_95_ values after 24 h of treatment (lethal concentration was designed to assess 50% and 95% of insect mortality).

### 2.8. Statistical Analysis

All data were expressed as means ± standard deviations of triplicate measurements. The confidence limits were set at *P* < 0.05. LC_50_ and LC_95_ were calculated by Probit analysis using IBM SPSS statistics version 19 (2010). Data were calculated for significance by ANOVA (one-way analysis of variance) using SPSS 20.1 (version IBM, 20.0.2004). Statistical differences between the essential oils were estimated by Tukey's test. Student's *t*-test analysis was used to compare between essential oil extraction yields. Multiple range tests were conducted at 5% significance level.

The article "Clove Buds Essential Oil: The Impact of Grinding on the Chemical Composition and Its Biological Activities Involved in Consumer's Health Security" was published in 2021. Journal: Biomed Res Int.

## 3. Results and Discussion

### 3.1. Extraction Yield

Obtained results showed that grounded samples (particle size = 0.6 mm) present the highest extraction yield. While the ungrounded clove buds (particle size between 1.5 and 2 cm) exhibited an EO extraction yield of 7.1 ± 0.8%, the grounded ones showed an extraction yield two times higher than the first EO and reached the value of 14.3 ± 0.6% (Figure 1). These results were in agreement with those found by Selles et al. [16] when working on the grounded buds of *S. aromaticum* essential oil from Algeria. They obtained an extraction yield of 11.6%. Similarly, Kapadiya and Desai [17] have found an extraction yield equal to 11.35% when the clove bud's particle size was about 565 microns. The current data showed the influence of the grinding method on the EO extraction yield, which is a technical practice, which enlarges the contact area between solid medium and the boiled water [18]. The decrease of particle size was related to the increase in essential oil extraction yield [17]. In addition, grinding improves the extraction speed and the hydrodistillation yield. However, extreme grinding may disturb the steam circulation, and thus slow down the extraction speed [19].

### 3.2. GC-MS Analysis

The volatile compounds of the different essential oils (grounded and ungrounded) of clove buds were analyzed by GC-MS (Figure 2). A comparison between the EO chemical composition obtained from grounded and ungrounded buds was elaborated. Results shown in Table 1 and Figures 2(a) and 2(b) indicate that eugenol was the major component for both ungrounded (87.4%) and grounded buds (68.7%). The current result was higher than that determined by Aguilar-González et al. [20], who found a peak area value of 75.4% for ungrounded clove buds. Cyperene ranks second with an average peak area of about 7.2 and 20.5%, respectively, for ungrounded and grounded clove buds. However, it was reported that *β*-caryophyllene (11.5%) was one of the major components [21]. This latter compound was not detected in this study. Furthermore, it was reported that eugenol, eugenol acetate, *β*-cariofilen, *α*-humulen, *β*-pinene, limonene, farnesol, benzaldehyde 2-heptanone, and ethylanoate were the most common compounds [21]. Accordingly, it was demonstrated that eugenol (75.4%) and caryophyllene oxide (11.2%) were the major compounds [20]. This variability in the extraction yield value and EO composition can be explained by the maturity stage and environmental factors (temperature, photoperiod, and hygrometry), the analytical methods, and the major effects of geographical and ecological variations among habitats [14]. The particle size has an effect on the extraction efficiency, which depends on the extraction conditions. Indeed, on the one hand, a decrease in the size of the particles will lead to an improvement in the specific surface area; the solvent, which is distilled water, penetrates more easily into the particles, thus increasing the quantity of EO and decreasing the internal transfer time of solutes. On the other hand, the process of grinding can lead indirectly to a decomposition of the plant material and thus to a reduction of the amount of volatile chemical compounds. These results are in accordance with those stipulated by Herzi [22]. Kapadiya and Desai [17] also indicated that size parameter is one of the most important factors influencing the essential oil extraction of clove buds. Their findings highlighted that the decrease of particle size involved an increase in the extraction yield and eugenol (10.30%), which was different from our results. In the current study, the amount of eugenol decreased with the grounding process, from 87.39% to 68.73%, respectively, for ungrounded and grounded clove bud essential oils; however, it is still much more higher than the values reported by Kapadiya and Desai [17] which is equal to eugenol at 10.36%. These differences could be related to the technical procedure, hydrodistillation time, heating, etc. In light of these results, one recommendation could be established. If the objective of the valorization is to have an essential oil concentrated in eugenol, the grinding procedure is not necessary. On the other hand, if the objective is to exploit the other active biomolecules, such as cyperene, *cis*-thujopsene, and phenyl isovalerate, it would be preferable to ground the clove buds to improve their contents in the obtained essential oil.

The article "Clove Buds Essential Oil: The Impact of Grinding on the Chemical Composition and Its Biological Activities Involved in Consumer's Health Security" was published in 2021. Journal: Biomed Res Int.

### 3.3. Antioxidant Activities: DPPH^•^ and FRAP Assays

Several researchers have reported the efficacy of employing DPPH radical and FRAP methods to evaluate the antioxidant potential by estimating the radical scavenging activity [23, 24]. Comparative evaluation of antioxidant potential of the different essential oils (grounded and ungrounded) of clove buds was established. Overall, clove essential oil is constituted of many powerful antioxidant components like eugenol, *β*-caryophyllene, and eugenyl acetate, which are known to inhibit reactive oxidative species by scavenging free radicals [6].  Figure 3 illustrates that the antioxidant activity of grounded bud EO (IC_50_ = 1.2 ± 0.1 *μ*g/mL) was about two times greater than that of ungrounded ones (IC_50_ = 2.8 ± 0.5 *μ*g/mL). These results were very significant when compared to BHT (IC_50_ = 35.5 ± 0.57 *μ*g/mL). These findings were in perfect agreement with Gülçin et al. [25] who reported that DPPH^•^ scavenging activity of clove bud EO was more important than various synthetic antioxidants, namely, BHT, *α*-tocopherol, and Trolox. This important activity could be related to the high content of eugenol according to many scientific reports proving that eugenol is a potent chelator with values of IC_50_, ranging from 4.4 to 130.5 *μ*g/mL [26, 27]. Results depicted in Figure 4 show that the efficiency concentration was dependent on clove bud particle size, which is a crucial parameter affecting the chemical composition as described in the previous section, and thus affecting the biological activities. In fact, when comparing this result to the one of chemical composition, we can deduce that the essential oil with the lower eugenol amount (68.73% for grounded clove buds) possesses a lower EC_50_ value (32 ± 1.3 *μ*g/mL) than theEC_50_value of intact buds (50 ± 4.5 *μ*g/mL) with eugenol amount of 87.39%.

The BHT EC_50_ was equal to 25.8 ± 0.2 *μ*g/mL in the same experimental conditions. This finding could be related to the loss and the decomposition of clove buds during the grinding process, and thus to a reduction of the amount of volatile chemical compounds. It is important to note that there are no previous citations concerning the FRAP test on clove buds EO. These results were obtained after three measurements for both clove batches (ungrounded and grounded).

### 3.4. Antibacterial Activity: Disc Diffusion Assay

Summarized results in Table 2 demonstrate that clove buds EO was very active against Gram^+^ and Gram^−^ bacteria with IZD ranging between 17.2 ± 4.5 and 35.5 ± 2.6 mm. Statistical analysis showed a significant difference between EO from grounded and ungrounded clove buds. These findings were in perfect agreement with previous reports which elucidated important MIC values for *L. monocytogenes* (0.05 mg/mL) and *S. enteritidis* (0.1 mg/mL) [28]. This activity could be attributed to the major compound “eugenol (>85%).” Indeed, it was demonstrated in an *in vitro* study that the MIC values of clove oil and eugenol to *Bacillus cereus* were 25 and 15 *μ*g/mL, and their MBC values were 40 and 25 *μ*g/mL, respectively, whereas the half maximal inhibitory concentration (IC_50_) of clove oil against this important food source gram-positive pathogen was 5.02 *μ*g/mL, and that of eugenol was 4.05 *μ*g/mL [29]. Radünz et al. [30] demonstrated that *S. aromaticum* EO containing 56.06% eugenol showed a strong inhibitory effect up to a concentration of 0.30 mg/mL against pathogenic bacteria (*E. coli* O157:H7, *L. monocytogenes*, and *S. aureus*) [30]. In addition, according to Thielmann et al. [31], *Syzygium aromaticum* revealed promising growth inhibitory activity with MICs of 100 and 400 *μ*g/mL, respectively, against *S. aureus* and *E. coli*. Abdullah et al. recorded an IZD against *S. aureus* of 13 ± 2.2 and 22 ± 1.6 mm at 1.3 and 10% concentration, respectively, [32]. However, antimicrobial activity cannot be attributed to the action of the major chemical component. Eugenol followed by aldehydes, ketones, and alcohols are the responsible compounds [33]. Besides, from Table 2, it is shown that *E. coli* is the most sensitive recording the highest IZD of about 28.7, 34, and 35.5 mm, respectively, to 1, 5, and 10 *μ*L applied doses. Besides, these results conventionally indicated that the increase of bioactive inhibitory power was closely correlated to EO type (from grounded or ungrounded buds) and concentration (Table 2). All these findings enhance the use of this spice as a natural food preservative and encourage its use in several fields: pharmaceutical, cosmetics, agriculture, and therapy. Indeed, eugenol besides other components such as *β*-caryophyllene and eugenol acetate [34, 35] has the main essential effects of clove as an anti-inflammatory, analgesic, antimicrobial, antiparasitic, antioxidant, antimutagenic, anticonvulsant, and anticarcinogenic agent [36, 37]. They are also known for their therapeutic potential to control vomiting, nausea, diarrhoea, flatulence, cough, and stomach distension; to relieve pain; and to cause uterine contraction [38]. All these biological activities contribute to the improvement of consumers' health. Clove EO has been found to show antifungal activity against pathogenic fungi, namely, *Tricophyton rubrum*, *Tricophyton mentagrophytes* var. *interdigitale*, *Epidermophyton flocosum*, *Candida* spp., and *Aspergillus* spp. [39, 40]. The antibacterial activity of clove EO alone and in combination with different antimicrobial compounds against common food-borne pathogens has been evaluated in a wide variety of food products such as cucumber [41], rainbow trout fillets [42], ground beef [43], cooked pork sausages [37], and ground chicken meat [44]. These findings allowed the application of this raw material as a natural bioconservative, as an alternative to synthetic ones, and thus preserving the wellbeing of consumers.

The article "Clove Buds Essential Oil: The Impact of Grinding on the Chemical Composition and Its Biological Activities Involved in Consumer's Health Security" was published in 2021. Journal: Biomed Res Int.

### 3.5. Allelopathic Effect

Figure 5 illustrates the *H. niger* germination rate under different clove buds EO concentrations. Noticeably better results were demonstrated for the essential oil (30 *μ*L) in comparison with the control seeds. Indeed, clove buds EO achieved complete inhibition of *H. niger* germination during the whole experiment period; however, only 91% was recorded for the control seeds. Controls prepared with a methanol/water (1‰) mixture did not affect *H. niger* germination in comparison with controls in water. In addition, obtained results showed the dose-dependent manner of the allelopathic effect. These findings were in line with those reported by Amparo-Blazquez [45], which indicated that *S. aromaticum* EO caused an important inhibition of seedling growth against broccoli, lambsquarters, and redroot pigweed. The mechanism of germination inhibition is not well known, but some studies reported that a lack of electrolyte, cell destruction, and membrane permeability caused by EO could be implicated [46]. An inhibition of water uptake in the plant cell, as well as some physiological and biochemical processes may also lead to germination inhibition [47]. EOs caused many changes in plant seedlings leading to reduction in some organelles, such as mitochondria and, in certain cases, inhibition of DNA synthesis [47]. These factors may explain the blockage of seed germination and embryo death. The application of eugenol on hybrid rice decreased its seed germination speed at 2 g/concentration [48]. Kegley et al. reported that the effectiveness of clove EO is only important as burnt herbicide used on growing plant leaves [49].

### 3.6. Insecticide Effect

The insecticidal activity was examined using the paper filter contact method. *S. oryzae* was significantly susceptible to the EO after 24 h of exposure. Probit analysis showed that 50% of mortality was achieved at 252.4 *μ*L/L air concentration, when the confidence limits were about 95%. LD_95_ was estimated at 426.2 *μ*L/L air. Cardiet et al. [50] mentioned that clove EO has an insecticidal activity against *S. oryzae* with LC_90_ observed at 355 *μ*L/L. According to Devi and Devi [51], *S. oryzae* was susceptible to the toxic effect of clove oil resulting in 92% mortality by 21 days. Vendan et al. [52] registered a44.90 ± 6.91%adult mortality in *S. oryzae* recorded at a concentration of 400 *μ*L/L air of clove oil and during 72 h of exposure time. Mishra et al. [53] reported that the essential oils extracted from *S. aromaticum* killed the adults of *S. oryzae* by fumigant action. They also mentioned that the fumigant toxicity was proportional to exposure time and concentration. The authors indicated that *S. aromaticum* EO had stronger toxicity in comparison to *A. marmelos* EO against *S. oryzae.* For that reason, Jairoce et al. [54] recommended clove bud EO as a promising alternative to be used under storage conditions for the integrated management of stored grains pest. Besides, Trivedi et al. [55] indicated that the LC_50_ value obtained for clove oil after 24 h exposure against *C. chinensis* adults was about 0.3 *μ*g/mL. The efficacy of clove oil is due to its major components, such as phenylpropanoids like carvacrol, thymol, eugenol, and cinnamaldehyde. The authors indicated that clove EO may be developed as possible natural fumigants or repellents to control the pulse beetle.

The article "Clove Buds Essential Oil: The Impact of Grinding on the Chemical Composition and Its Biological Activities Involved in Consumer's Health Security" was published in 2021. Journal: Biomed Res Int.

## 4. Conclusion

The main objectives of this study were the chemical and biological evaluations of *S. aromaticum* essential oil. The assessment of the grinding effect on clove buds EO was performed initially. It was demonstrated that the grounded buds gave higher essential oil yield than intact ones, with respective values of 14.3 and 7.1%. Chemical composition analysis identified particularly four major compounds, respectively, as mentioned below for unground and ground clove buds EOs: eugenol (87.4-68.7%), cyperene (7.2-20.5%), phenethyl isovalerate (3.6-6.4%), and *cis*-thujopsene (0.8-1.9%). *α*-Patchoulene was present at 0.2% in the chemical composition of grounded clove bud EO. For the antibacterial activity, the best inhibition zone diameter was observed against *E. coli*(35.5 ± 2.6 mm), when the grounded clove buds EO was applied. This important antimicrobial activity enhances the potential use of essential oil as a food preservative. Regarding the antioxidant power, both tested EOs were more potent radical DPPH scavengers (IC_50_ values of 2.8 ± 0.5 and 1.2 ± 0.1 *μ*g/mL, respectively, for ungrounded and grounded buds) than *α*-tocopherol, as they exhibited noticeable ferric-reducing power (EC_50_ = 32 and 50 *μ*g/mL, respectively, for intact and grounded clove buds). The significant antioxidant power encourages the application of clove buds essential oil in the composition of several drugs as a natural remedy. Furthermore, our results highlighted the potent herbicidal effect of *S. aromaticum* oil on seed germination of *H. niger*, as well as its allelopathic effect. These findings promote the use of clove buds essential oil as a synthetic pesticide alternative to preserve maize, wheat, or other grass seeds during their storage period.

## Figures and Tables

**Figure 1:** Extraction yield from grounded and ungrounded clove buds essential oil (%).

**Figure 2:** GC-MS chromatograms of (a) grounded and (b) ungrounded clove buds essential oils. (1) Eugenol; (2) cyperene; (3) *cis*-thujopsene; (4) phenethyl isovalerate.

**Figure 3:** The antioxidant activity of clove buds essential oil expressed as IC_50_ (*μ*g/mL) using the free radical scavenging capacity by DPPH assay compared to a standard BHT.

The article "Clove Buds Essential Oil: The Impact of Grinding on the Chemical Composition and Its Biological Activities Involved in Consumer's Health Security" was published in 2021. Journal: Biomed Res Int.

**Figure 4:** The equivalent reducing power from different samples of clove buds essential oil compared to the standard BHT expressed as EC_50_ (*μ*g/mL).

**Figure 5:** The germination percentage of *H. niger* decreased in a dose-dependent manner in the presence of grounded clove buds essential oil.

**Table 1:** Chemical composition of *S. aromaticum* essential oil extracted from ungrounded and grounded clove buds.

Compounds	RT_C_	RI_C_	RI_L_	% peak area of the chemical component	
				Ungrounded buds	Grounded buds
Eugenol	15.83-15.96	1344	1351 [56]	87.39	68.73
Cyperene	17.31	1396	1398 [57]	7.22	20.52
*cis*-Thujopsene	18.02-18.10	1427	1426 [58]	0.75	1.94
Phenethyl isovalerate	19.82-19.83	1498	1495 [59]	3.63	6.41
Total identified compounds				98.99	97.77
Phenolic compounds				87.39	68.73
Sesquiterpenes				7.97	22.63
Others				3.63	6.41

RI_C_: calculated retention index of the chemical compound; RT_C_: calculated retention time; RI_L_: retention index from literature.

**Table 2:** Antimicrobial activity of clove buds essential oil.

Doses (*μ*L)/strains	EO from (grounded buds)			EO from (ungrounded buds)			Antibiotics			
	1	5	10	1	5	10	GM	C	E	P
Diameter of inhibition zone (mm)										
*B. cereus*	27.3 ± 4.9^a^	29.0 ± 3.2^a^	32.1 ± 4.0^a^	22.3 ± 1.6^a^	26.3 ± 2.4^a^	29.0 ± 5.0^a^	—	—	25 ± 0^a^	—
*S. aureus*	29.5 ± 6.5^a^	30.0 ± 2.7^a^	32.0 ± 3.6^a^	21.6 ± 1.4^a^	25.3 ± 5.3^a^	26.5 ± 4.0^a^	—	—	—	38 ± 2^a^
*L. monocytogenes*	28.0 ± 5.6^a^	29.8 ± 1.0^a^	31.5 ± 3.7^a^	17.2 ± 4.5^b^	20.3 ± 4.3^b^	21.6 ± 2.1^b^	24 ± 0^b^	—	—	—
*E. coli*	28.6 ± 1.4^a^	34.0 ± 3.5^a^	35.4 ± 2.6^a^	26.0 ± 3.2^b^	26.8 ± 1.6^b^	28.0 ± 1.6^b^	—	30 ± 1^a^	—	—
*S. enteritidis*	25.8 ± 1.2^b^	28.5 ± 1.8^b^	29.6 ± 3.3^b^	21.4 ± 3.1^c^	22.2 ± 1.9^c^	25.0 ± 3.7^c^	—	—	36 ± 2^a^	—

The different superscripts in the same line means significant difference (*P* ≤ 0.05). All antibiotics were applied at a concentration of 0.33 *μ*g/mL. GM: gentamicin; C: chloramphenicol; E: erythromycin; P: penicillin. Pure essential oil was applied on a surface of 6 mm disc.

## Data Availability

The datasets generated during the current study are available from the corresponding authors upon reasonable request.

## Abbreviations

ATCC: American Type Culture Collection
BHT: Butylated hydroxytoluene
C: Chloramphenicol
DPPH: 2,2-Diphenyl-1-picrylhydrazyl
E: Erythromycin 500
EO: Essential oil
FeCl_3_: Iron chloride (III)
FRAP: Ferric-reducing antioxidant power
GC-MS: Gas chromatography-mass spectrometry
GM: Gentamicin
IP: Inhibition percentage
IZD (*Ф*): Inhibition zone diameter
K_3_Fe (CN)_6_: Potassium ferricyanide solution
MBC: Minimum bactericidal concentration
MIC: Minimum inhibitory concentration
Na_2_SO_4_: Anhydrous sodium sulfate
NIST: National Institute of Standards and Technology
P: Penicillin
RI: Retention index
TCA: Trichloroacetic acid.
